# Application of PET Imaging in the Brain Regions of the Emotional Control Loop in Patients with Generalized Anxiety Disorder

**DOI:** 10.1155/2021/4505227

**Published:** 2021-07-22

**Authors:** Jing Li, Wenjun Ouyang

**Affiliations:** ^1^Hubei Provincial Hospital of Traditional Chinese Medicine, Wuhan 430000, China; ^2^School of Economics and Management, China University of Geosciences (Wuhan), Wuhan 430000, China

## Abstract

**Objective:**

This study uses PET imaging to observe the uptake and metabolism of 18F-fluorodeoxyglucose (^18^F-FDG) in the multibrain areas of the emotional control loop in patients with generalized anxiety disorder (GAD) and investigate the brain of GAD patient's functional abnormality mechanism.

**Methods:**

The thesis clinically collected 20 GAD patients and 20 healthy subjects. Dynamic PET-CT scans were used. At the same time, ^18^F-FDG whole-brain uptake and metabolism data were collected. Image fusion and semiquantitative analysis were used to measure emotional control loops. The maximum standard uptake value (SUVmax) and dynamic uptake and metabolic changes of 11 time points in the brain area at 150 min were measured.

**Results:**

Compared with the healthy control group, the peak uptake of the bilateral prefrontal cortex and the average uptake rate before the peak in GAD patients were significantly reduced (*P* < 0.05), and the average metabolic rate after the peak was significantly increased (*P* < 0.05). The peak uptake of the left striatum and the left hippocampus, the average uptake rate before the peak, and the average metabolic rate after the peak were all significantly reduced (*P* < 0.05); There were no obvious changes in the three indexes of the right striatum and the right hippocampus.

**Conclusion:**

There are ^18^F-FDG uptake and metabolic disorders in multiple brain areas of the affective control loop of GAD patients. The abnormal peak and rate of uptake may be related to the pathogenesis of GAD.

## 1. Introduction

Generalized Anxiety Disorder (GAD) is a common mental illness. Patients have emotional disorders such as anxiety, tension, and fear, which often seriously affect normal life. Research on the pathogenesis of GAD is currently mostly focused on the fields of neurotransmitter and brain structure and function, and there are few studies from the level of molecular imaging. 18F-Fluorodeoxyglucose (^18^F-FDG) PET-CT imaging is a technology that has been gradually used in clinical work in recent years. It can reflect the degree of somatic cell activity from the side, especially in the research of central nervous disease. The level reflects the function of nerve cells. At present, it has been well used in many fields such as stroke, brain tumor, and Alzheimer's disease and can accurately determine the distribution, range, and degree of nerve cell activity [1, 2]. There are many abnormalities in GAD, such as atrophy of gray matter nuclei in the brain area of the affect-regulated brain area, functional link disorder of the brain area, and neurotransmitter imbalance. These abnormal changes affect and interact with each other, and the pathogenesis is very complicated. Based on whole-brain imaging, this study dynamically observed the ^18^F-FDG uptake and metabolism characteristics of nerve cells in the brain area of the emotional control loop and provided an objective basis for abnormal information interaction feedback and regulatory disorders in each brain area to supplement and improve the pathogenesis of GAD.

## 2. Materials and Methods

### 2.1. Clinical Data

The thesis collected 20 GAD patients in the neurology clinic of our hospital. All patients included 9 males and 11 females, aged 21 to 58 years, with an average of 33.9 ± 3.4 years; the patient's years of education were 9–16 (14.5 ± 3.5) years; height was 150～179 (155 ± 12) cm; weight 47～82 (60 ± 11) kg; and all patients were right handed [3, 4]. Conditions for patients to enter the group: (1) they all met the GAD diagnostic criteria of the Chinese Classification and Diagnostic Criteria for Mental Disorders 3rd Edition (CCMD3) and Hamilton Anxiety Scale (HAMA) score ≥ 14 points; (2) head MRI excludes brain organic diseases or development abnormality; (3) clinical-scale evaluation excludes depression, schizophrenia, and other mental diseases; and (4) not recently (within 3 months) taking hormones, antianxiety, and other psychotropic drugs that affect glucose intake.

Taking the staff of the hospital and their families as sources, this study collected a total of 20 cases in the healthy control group. There were 9 males and 11 females in the healthy group, aged 23 to 60 years, with an average of 35.3 ± 3.7 years; the years of education in the group were 9–19 (15.4 ± 2.7) years; height was 155–180 (160 ± 10) cm; weight was 41–79 (56 ± 9) kg; and all were right handed. Inclusion criteria: (1) clinical-scale evaluation to exclude any mental illness; (2) head MRI to exclude brain organic diseases or developmental abnormalities; and (3) recently (within 3 months), no drugs that affect glucose uptake have been taken.

### 2.2. PET-CT Image Acquisition

Preparations before and during the scan: the subject started smoking and alcohol prohibition 1 day before the examination, avoiding the intake of drinks such as coffee, strong tea, and sugar water, sitting still for half an hour before the scan, closing the eyes during the scan, and trying to keep calm breathing. The study used a SIEMENS52 ring 128-layer high-resolution PET-CT scanner; the imaging agent ^18^F-FDG was produced by Canada's EBCOTR19 medical cyclotron, with radiochemical purity >95%. The data collection method is as follows: after the subject's measured blood glucose reaches the target, they will be injected with ^18^F-FDG intravenously, the total amount of injection = body weight (kg) × 0.1 mCi, and keep calm for 10 minutes. All of them first performed CT head scan for anatomical positioning and then used the dynamic list mode to collect PET data at 11 time points at an interval of 15 minutes [5]. The data are reconstructed by the iterative method after attenuation correction and processed in the syngo True DVE12A workstation to obtain multiplanar reconstruction images.

### 2.3. A Semiquantitative Analysis of the Region of Interest of ^18^F-FDG Uptake in the Emotional Regulation Brain Area

Because the CT anatomy of the brain tissue is fuzzy and the accuracy is not good, the subjects in this study have been examined by the head MRI before being enrolled. Based on the 3D-T1WI sequence of the same subject, a multiresolution nonparametric density model was used (MRNDM), image fusion method, which transforms the RGB space of the source multimodal medical image registration into a generalized intensity-hue-saturation space (GIHS). Then, the MRI brain image of the patient is decomposed into low- and high-frequency components using nonsubsampled contour transformation (NSCT), and the fusion image is constructed by inverse operation of the NSCT operation of all composite coefficients. This method effectively overcomes the problem of model mismatch and can provide an accurate anatomical positioning basis for the outline of the region of interest [6]. The outline of the region of interest based on the ALL template and the anatomical landmark points of each brain area proposed by Ax macher, respectively, outlines the prefrontal cortex, striatum, hippocampus, and thalamus in the emotional control brain area. After the region of interest is delineated, the highest dynamic standard uptake value (SUVmax value, unit of Bq/cc) of ^18^F-FDG in the region is measured, and the data are automatically generated by the PET workstation software. The data of each point of 11 time points measured in each brain area were measured 3 times and averaged. Since ^18^F-FDG uptake and metabolism in the cerebellar region are recognized as relatively stable, the SUVmax value of the ipsilateral cerebellar structure of the same subject was standardized based on SUVmax (standardized) = SUVmax (brain area of interest)/SUVmax (same as the lateral cerebellum). The ^18^F-FDG peak value (the highest value of SUVmax in all time points), the average uptake rate before the peak, and the average metabolic rate after the peak of the brain area of interest were recorded. Average uptake rate before peak = [SUVmax peak − SUVmax (time starting point)]/peak time and average metabolic rate after peak = [SUVmax peak − SUVmax (time end point)]/postpeak time were recorded. Finally, Graph Pad Prism software was used to draw the time dynamic curve.

### 2.4. Statistical Analysis

Using SPSS11.0 software for statistical analysis, the data obtained in the experiment accord with the normal distribution, and the measurement data are expressed as mean ± standard deviation. A two-sample *t*-test was used to compare the two groups, and *P* < 0.05 indicated that the difference was statistically significant [7].

Context Awareness (CA) is a visual saliency model based on the contrast method. It uses LAB color space features to calculate the distance between two pixel blocks and define dissimilarity and then calculate the contrast of the 64 nearest neighbors of the current block; finally, feature maps such as color and distance are merged, and context correction and enhancement are performed to obtain a saliency map. The context-aware model follows the four criteria of bottom-level features, global features, organizational rules, and high-level elements. Among them, the first three points are calculated by color mode difference, global feature universality, and the relative concentration of salient feature pixels to calculate the salient area [8]. Finally, this paper adds feature elements to postprocess the salient map. The specific steps and calculation formula are as follows.

We divide the target image into *n* × *n* blocks and calculate the Euclidean color distance and the Euclidean space distance of the two pixel blocks in the LAB space, denoted by *d*_color_(*p*_*i*_, *p*_*j*_) and *d*_position_(*p*_*i*_, *p*_*j*_), respectively. Among them, *p*_*i*_ and *p*_*j*_ represent pixel block *i* and pixel block *j*. The saliency of a pixel block is jointly determined by *d*_color_(*p*_*i*_, *p*_*j*_) and *d*_position_(*p*_*i*_, *p*_*j*_). The larger the color distance and the smaller the position distance, the greater the difference between the two pixel blocks. The pixel block dissimilarity calculation formula is

(1) $$\begin{array}{c} D\left(p_{i},p_{j}\right)=\frac{d_{\text{color}}\left(p_{i},p_{j}\right)}{1+c\times d_{\text{position}}\left(p_{i},p_{j}\right)}. \end{array}$$

Here, *c* is a constant. Taking the saliency value of the pixel block pi as an example, the greater the difference between *p*_*i*_ and the surrounding pixel blocks, the higher the saliency. The reference set is {*q*_*k*_}_*k*=1_^*K*^. *K* = 64 is the number of selected pixel blocks, calculated as

(2) $$\begin{array}{c} S_{i}^{r}=1-\exp\left\{-\frac{1}{K}\sum_{k=1}^{K}d\left(p_{i}^{r},q_{k}^{r}\right)\right\}. \end{array}$$

Equation (2) can be used improve the contrast between the salient area and the insignificant area by taking the average value. The calculation formula is

(3) $$\begin{array}{c} S_{i}^{r}=1-\exp\left\{-\frac{1}{K}\sum_{k=1}^{K}d\left(p_{i}^{r},q_{k}^{rk}\right)\right\}. \end{array}$$

The range of saliency value is [0,1]; the larger the two pixel blocks, the higher the saliency and the smaller the less significant for pixels around salient points. The paper needs to add context for correction, by setting the saliency threshold and calculating the Euclidean distance weighted value between the salient point and the surrounding pixels to obtain the saliency value of the information [9]. After the thesis is revised, the saliency value of the salient area is enhanced. The context correction calculation method is shown as follows:

(4) $$\begin{array}{c} {\hat{S}}_{i}={\bar{S}}_{i}\left(1-d_{\text{foci}}\left(i\right)\right),\;{\bar{S}}_{i}=\frac{1}{M}\sum_{r\in R}S_{i}^{r}. \end{array}$$

After the target image is processed as mentioned above, a two-dimensional saliency map with the same size as the original image is obtained, as shown in Figure 1.

Grab cut characterizes the probability distribution of color information by estimating the Gaussian Mixture Model (GMM) of the target area and the background area. On the RGB space color image, the pixel GMM Gaussian component is allocated, the parameters are optimized, and the segmentation prediction is iterated to converge to obtain the foreground area. Finally, the paper uses the smoothest boundary of the foreground area to improve the edge accuracy of the segmented image [10].

The Grab Cut algorithm requires user initialization to divide the target image into a background area and possible target areas. The pixels in the two areas are initialized to 0 and 1, respectively [11]. The pixel point set *a*=(*a*_1_,…*a*_*n*_,…, *a*_*N*_), *a*_*n*_ ∈ {0,1} corresponds to the pixel point label set *K*=(*k*_1_,…*k*_*n*_,…, *k*_*N*_). Among them, *N* is the number of pixels; *θ* is the color probability distribution model of the target area and the background area; and *K* is the number of Gaussian distribution (*K* = 5). The problem is described as follows:

(5) $$\begin{array}{c} a=\arg\underset{a}{\min}E\left(a,\theta \right). \end{array}$$

The Gibbs energy used by Grab Cut on the RGB space color image is

(6) $$\begin{array}{c} E\left(\underline{a},k,\underline{\theta },z\right)=U\left(\underline{a},k,\underline{\theta },z\right)+V\left(\underline{a},z\right). \end{array}$$

Here, *E* is the Gibbs energy, *U* is the data item, *V* is the smooth item, and *z* is the image gray value array, *z*=(*z*_1_,…*z*_*n*_,…, *z*_*N*_). The parameters of the Gaussian mixture model are

(7) $$\begin{array}{c} \underline{\theta }=\left\{\pi \left(a,z\right),u\left(a,k\right),\sum \left(a,k\right)\right\}. \end{array}$$

Here, *a*=0, *k*=1,…, *K*. The boundary energy term *V* is solved using the Euclidean distance formula in the RGB space:

(8) $$\begin{array}{c} V\left(\underline{a},z\right)=y\sum_{\left(m,n\right)\in C}\left[a_{n}\neq a_{m}\right]\exp-\beta {\left\|z_{m}-z_{n}\right\|}^{2}. \end{array}$$

Here, *m* and *n* represent two neighborhood pixels; the value of parameter *β* is inversely proportional to the contrast of the image, so that the boundary energy term *V* can be applied to high-contrast and low-contrast images; and the constant *γ* is obtained from image training. This paper uses this method to obtain a segmentation curve with smooth edges, as shown in Figure 2.

## 3. Results

### 3.1. The Distribution of Abnormal Uptake in the Emotional Control Loop

F-FDGPET-CT imaging showed that the whole-brain uptake distribution of the GAD group and healthy control group was clear. Compared with the healthy control group, the peak uptake of the bilateral prefrontal cortex and the average uptake rate before the peak in the GAD group were significantly reduced (*P* < 0.05), and the average metabolic rate after the peak was significantly increased (*P* < 0.05); the peak uptake in the lateral striatum and the left hippocampus, the average uptake rate before the peak, and the average metabolic rate after the peak were all significantly reduced (*P* < 0.05); the peak uptake in the left thalamus, the average uptake rate before the peak, and the peak average metabolic rate after the peak increased significantly (*P* < 0.05); and the peak uptake in the right thalamus and the average uptake rate before the peak increased significantly (*P* < 0.05), and there was no significant difference in the average metabolic rate after the peak [12]. There were no obvious changes in the three indexes of the right striatum and the right hippocampus. The specific data in the paper are shown in Tables 1–3.

### 3.2. Dynamic Characteristics of Abnormal Uptake in the Brain Area of the Emotional Control Loop

Compared with the healthy control group, during the ^18^F-FDG imaging process, the GAD group showed slow advancement and faster delivery and decreased total amount on both sides of the prefrontal cortex; the left striatum showed slow advancement and slow exit and decreased total amount. There was no significant difference in changes in the lateral striatum; the left hippocampus showed slow entry and slow exit, and the total amount decreased, and the right hippocampus showed no significant difference; the left thalamus showed fast forward and faster exit, and the total amount increased, the right thalamus showed fast in and out, and the total volume increases performance [13] (see Figures 3 and 4).

## 4. Discussion

GAD has a number of functional abnormalities in brain structures, and the dysfunction of the affect regulation loop is a key factor leading to the disease. Structural magnetic resonance studies have shown that the prefrontal cortex, striatum, hippocampus, and thalamus contained in this loop have varying degrees of morphological abnormalities. The main manifestations are the reduction of brain volume and the reduction of gray matter thickness; functional magnetic resonance is here on the basis of this, and it is further confirmed that there are abnormal functional linkages between multiple brain areas of the emotional control loop. For example, there is an increase in the activation of the thalamus and the hippocampus, the prefrontal cortex, and the decrease of the activation of the hippocampus and the prefrontal cortex while the brain structure is atrophy [14]. Conventional MRI technology can certainly observe and explore the mechanism of GAD imaging performance to a certain extent, but due to differences in data collection, correction, and normalization steps, there are still many differences and controversies in the final results, and MRI lacks dynamic brain function. Technical means of change observation.

F-FDGPET-CT, as a new technology for observing changes in brain nerve cell function in recent years, can clearly visualize the glucose uptake and metabolism process of nerve cells. This technology presents brain function changes in image data through the dynamic acquisition mode, which can compensate for MRI observation of the cell metabolism process that is difficult to achieve in brain function research, realizing the real molecular imaging level research. GAD patients have significant mental disorders such as anxiety, tension, and fear, and the nerve cells in the brain area of the emotional control loop have a significantly different demand for glucose energy from healthy people [15].

The results of this study showed that the peak uptake of the bilateral prefrontal cortex in GAD patients decreased and the average uptake rate before the peak decreased, which was consistent with the results of PET experiments in rat models of other scholars, but the time gradient results suggested that the brain area was average after the peak. The metabolic rate is significantly accelerated; the peak uptake of the hippocampus and striatum on the left side decreases, and the average postpeak metabolic rate slows down, similar to the results of the literature; our results also show that the peak uptake of the bilateral thalamus increases, reaching the prepeak The average uptake rate increases, and the average metabolic rate after the left thalamic peak increases [16]. Dynamic analysis of abnormal ^18^F-FDG uptake in various brain regions shows that, in the emotional regulation loop of GAD patients, the thalamus structure, which is a rough information processing area, has a significant increase in the demand for glucose energy and the use of conversion rate is accelerated, as a fine information adjustment transmission The hippocampus and striatum in the central part of the hippocampus and striatum have a significant insufficient demand for glucose energy and a tendency to stagnate conversion. The prefrontal cortex, which has information executive functions, has insufficient demand for glucose energy but uses it to transform too quickly [17]. The possible mechanism for the occurrence of this misaligned energy demand and application inequality is that, with the continuous increase in external stress events, sensitive individuals absorb too many negative stimuli, resulting in a certain degree of regulatory transmission dysfunction.There are insufficient executive functions, unable to adapt and deal with too many adverse events, and there are also obstacles to the feedback implementation of benign regulation, which are prone to anxiety and fear-like behaviors and eventually lead to the occurrence of GAD. For the right emotional regulation loop, the study only shows abnormalities in the thalamus and prefrontal cortex, and the intermediate regulatory transmission center is not affected. In addition to the theory of the dominant hemisphere of the brain, the thesis needs to further study its mechanism.

## 5. Conclusions

To sum up, there are abnormalities in ^18^F-FDG uptake and metabolism in multiple brain regions in the nutriregulation circuit of GAD patients. Abnormal uptake peaks and rates may be related to the onset of GAD. Dynamic observation of its changes can help reveal deeper the pathogenesis of GAD.

## Figures and Tables

**Figure 1:** Two-dimensional saliency map of brain PET.

**Figure 2:** Segmentation curve with smooth edges.

**Figure 3:** ^18^F-FDG imaging of the bilateral prefrontal cortex showed slow advance and fast exit, and the total amount decreased.

**Figure 4:** The left striatum of ^18^F-FDG showed slow in and slow out, and the total amount decreased.

**Table 1:** The difference of the peak uptake of the two groups of emotional control loops in multiple brain regions (Bq/cc).

Grouping	Left prefrontal cortex	Right prefrontal cortex	Left striatum	Right striatum	Left hippocampus	Right hippocampus	Left thalamus	Right thalamus
Healthy control group	2.41 ± 0.21	2.52 ± 0.24	1.95 ± 0.17	1.97 ± 0.22	1.65 ± 0.20	1.63 ± 0.19	1.71 ± 0.17	1.69 ± 0.15

GAD group	2.04 ± 0.20	2.06 ± 0.18	1.41 ± 0.19	1.97 ± 0.18	1.16 ± 0.15	1.63 ± 0.16	2.13 ± 0.24	2.08 ± 0.20

*t* value	5.71	6.86	9.47	0	8.77	0	6.39	6.98

*P* value	<0.05	<0.05	<0.05	>0.05	<0.05	>0.05	<0.05	<0.05

**Table 2:** The difference in the average uptake rate of the two groups of emotional control loops before the peak of the multibrain area [Bq/(cc·min)].

Grouping	Left prefrontal cortex	Right prefrontal cortex	Left striatum	Right striatum	Left hippocampus	Right hippocampus	Left thalamus	Right thalamus
Healthy control group	0.34 ± 0.02	0.24 ± 0.02	0.14 ± 0.01	0.09 ± 0.01	0.12 ± 0.02	0.11 ± 0.02	0.21 ± 0.02	0.08 ± 0.01

GAD group	0.15 ± 0.01	0.15 ± 0.02	0.09 ± 0.01	0.09 ± 0.01	0.06 ± 0.01	0.11 ± 0.01	0.45 ± 0.03	0.14 ± 0.01

*t* value	38	14.23	15.81	0	12	0	29.77	18.97

*P* value	<0.05	<0.05	<0.05	>0.05	<0.05	>0.05	<0.05	<0.05

**Table 3:** Differences in the average metabolic rate of the two groups of emotional control loops after peaking in multiple brain regions [Bq/(cc·min)].

Grouping	Left prefrontal cortex	Right prefrontal cortex	Left striatum	Right striatum	Left hippocampus	Right hippocampus	Left thalamus	Right thalamus
Healthy control group	0.07 ± 0.01	0.05 ± 0.02	0.08 ± 0.01	0.12 ± 0.02	0.09 ± 0.01	0.11 ± 0.02	0.05 ± 0.01	0.10 ± 0.01

GAD group	0.10 ± 0.01	0.12 ± 0.02	0.03 ± 0.01	0.11 ± 0.02	0.05 ± 0.01	0.10 ± 0.01	0.08 ± 0.01	0.09 ± 0.02

*t* value	9.49	11.07	15.81	1.58	12.65	2.1	9.49	2.1

*P* value	<0.05	<0.05	<0.05	>0.05	<0.05	>0.05	<0.05	>0.05

## Data Availability

The data used to support the findings of this study are available from the corresponding author upon request.
